# Dengue Risk Forecast with Mosquito Vector: A Multicomponent Fusion Approach Based on Spatiotemporal Analysis

**DOI:** 10.1155/2022/2515432

**Published:** 2022-06-02

**Authors:** Linlin Li, Zhiyi Fang, Hongning Zhou, Yerong Tang, Xin Wang, Geng Liang, Fengjun Zhang

**Affiliations:** ^1^College of Computer Science and Technology, Jilin University, Changchun, China; ^2^Institute of Software, Chinese Academy of Sciences, Beijing, China; ^3^Yunnan Institute of Parasitic Diseases, Puer, China; ^4^State Key Laboratory of Computer Science, Institute of Software, Chinese Academy of Sciences, Beijing, China

## Abstract

Dengue as an acute infectious disease threatens global public health and has sparked broad research interest. However, existing studies generally ignore the spatial dependencies involved in dengue forecast, and consideration of temporal periodicity is absent. In this work, we propose a spatiotemporal component fusion model (STCFM) to solve the dengue risk forecast issue. Considering that mosquitoes are an important vector of dengue transmission, we introduce feature factors involving mosquito abundance and spatiotemporal lags to model temporal trends and spatial distributions separately on the basis of statistical properties. Specifically, we conduct multiscale modeling of temporal dependencies to enhance the forecast capability of relevant periods by capturing the historical variation patterns of the data across different segments in the temporal dimension. In the spatial dimension, we quantify the multivariate spatial correlation analysis as additional features to strengthen the spatial feature representation and adopt the ConvLSTM model to learn spatial dependencies adequately. The final forecast results are obtained by stacking strategy fusion in ensemble learning. We conduct experiments on real dengue datasets. The results indicate that STCFM improves prediction accuracy through effective spatiotemporal feature representations and outperforms candidate models with a reasonable component construction strategy.

## 1. Introduction

Dengue is an acute infectious disease transmitted by mosquito vectors that cause flu-like symptoms and can be fatal [1]. According to World Health Organization (WHO) estimates, 40% of the world's regions are exposed to dengue risk. About 50-100 million people are infected with dengue each year, including up to 500,000 life-threatening cases of dengue shock syndrome [2]. Dengue poses a continuous threat to global public health and has become one of the new infectious diseases in China. In the absence of an effective vaccine against dengue, the impact of responses as cases occur on the epidemic is limited and valid methods are urgently required to forecast dengue outbreak risks.

The current dengue-related forecast models utilize similar characteristic parameters, generally only considering the case sequence and meteorological factors [3]. However, dengue is transmitted by mosquitoes in actual scenarios, and its risk forecast requires considering the direct impact of mosquito vector abundance. As the dengue vector, *Aedes* mosquitoes carry on the spread primarily rely on *Aedes aegypti* and *Aedes albopictus* [1]. Their reproduction precedes disease transmission, and inhibition in its immature stage would alleviate the pressure of disease outbreaks. Vector surveillance quantitatively measures the number and distribution of mosquitoes by investigating their breeding environment. Larval indices as a favorable candidate for interpreting mosquito vector density can be considered a predictor of dengue risk [4]. But apart from utilizing larval indices as features to construct forecast models [5], the application of the correlation quantification between dengue cases and mosquito abundance in the risk forecast of mosquito-borne infectious diseases remains limited, especially in the spatial dimension [6, 7].

In practical forecast scenarios, it is crucial to explore spatiotemporal correlations between dengue cases and larval indices by constructing data contexts embedded in continuous space and vary dynamically over time [8]. Specifically, it is to learn static attribute features and dynamic spatiotemporal features with a global perspective.  Figure 1 visualizes the spatiotemporal correlation between dengue risk and mosquito abundance. The horizontal direction denotes three time slices, each covering five nodes in the spatial dimension, where nodes within adjacent grids are considered neighbors. The yellow line indicates the temporal dependence of the node at the current moment on historical moments. The blue line indicates the spatial dependence of the node on the adjacent nodes at the same time. The red line indicates the spatiotemporal dependence of the node at the current moment on adjacent nodes at historical moments. Mining crux features and accurately forecasting dengue risk from such complex multivariate spatiotemporal data remain exploratory. There are still issues not fully resolved by existing research works, which are summarized as follows:

- *I*_1_*: Multiscale Analysis of Historical Variations in Dengue Risk and Mosquito Vectors*. Some studies analyzed temporal correlations between entomological indicators and dengue cases as mosquito abundance exhibits weather-influenced seasonal variation and induces disease [4, 9, 10]. Analyzing the historical variation patterns of time series can obtain valuable information, but most existing studies consider adjacent historical segments. Given long-term trends and short-term anomalies reflect temporal variations from different perspectives, a multiscale analysis of history should be considered
- *I*_2_*: Explaining the Geographic Distribution of Dengue Risk by the Spatial Cluster Pattern of Mosquito Vectors*. In addition to the analysis of environmental factors, the existing spatial modeling methods of mosquito vector density mainly involve the exploration of spatial aggregation but only cover the range of spatial autocorrelation [11]. Specifically, the local Moran's index serves as a spatial autocorrelation metric to explore local changes in spatial aggregation by measuring the relative contribution of variables in each region [12]. Evidence for the spatial correlation between dengue cases and mosquito abundance is still lacking
- *I*_3_*: Introduce Spatiotemporal Correlation Factors into Predictive Models*. Due to the spatiotemporal properties of dengue transmitted by mosquitoes, the assessment strategy to investigate the association between dengue risk and mosquito abundance from both temporal and spatial dimensions is a requisite consideration for studying dengue dynamics. Multivariate spatiotemporal correlations have the potential to be feature factors in dengue risk forecast models, but the availability has not been further validated. To bridge this research gap, this work introduces spatiotemporal correlation factors into the dengue risk forecast task and verifies the effectiveness of its mathematical metrics in the prediction model

By jointly considering the above issues, we propose a multicomponent fusion forecast approach based on multivariate spatiotemporal analysis, STCFM. It analyzes the temporal-lag cross-correlation of dengue risk and larval indices and simultaneously explores the binary expansion of spatial autocorrelation, i.e., multivariate spatial correlation. The spatiotemporal correlation metrics are further introduced into the dengue risk forecast model. Empirical studies indicate STCFM boosts performance and provides crux spatiotemporal features for forecast. The specific contributions of this paper are summarized as follows:

- We utilized the temporal lag cross-correlation function to analyze the mathematical association between dengue risk and larval indices and constructed multiscale features at different time intervals (addressing *I*_1_). By capturing the short-, mid-, and long-period variation patterns of time series, it can more comprehensively depict the periodicity characteristics and build the component model for prediction (addressing *I*_3_)
- Considering the nature of dengue risk and larval indices as spatiotemporal data, we conducted a spatial analysis of temporal data containing geographic information. Specifically, we exploit the multivariate domain expansion of local spatial autocorrelation to explore the impact of the spatial cluster pattern of mosquito vectors on the dengue transmission region (addressing *I*_2_) and introduce the correlation indicator as an additional feature into the spatial component model (addressing *I*_3_)
- We train a fusion model involving spatiotemporal components on a real dengue infectious disease dataset to verify the performance. Empirical results show that STCFM outperforms other candidate models, and both the temporal and spatial components can efficaciously improve the forecast consequence

## 2. Related Work

Time series forecast in epidemiology has a broad discussion involving multivariate feature extraction and diverse prediction models. Existing models have demonstrated competitiveness in disease risk forecast, albeit with different tasks and characteristics. Considering disease transmission exhibits spatiotemporal dependence, we have the following two concerns for disease risk forecast models based on spatiotemporal analysis.

### 2.1. Forecast Models

Statistical analysis approaches and deep learning algorithms are widely adopted in time series forecasting. Statistical analysis approaches such as Autoregressive Integrated Moving Average (ARIMA) validate the significance of inferences by analyzing associations among variables, focusing on the analytical process. Deep learning algorithms are specialized in mining rules from historical data for prediction instead of hypothesis testing in statistical models to demonstrate statistical significance. These include feedforward neural networks (FNN), recurrent neural networks (RNN), and convolutional neural networks (CNN). Statistical analysis approaches for dynamic forecast of disease risks are difficult to capture seasonal patterns and irregular variations simultaneously, and deep learning algorithms have obvious advantages in this regard [3, 13]. Some research works combine statistical analysis approaches and deep learning algorithms to provide fruitful solutions, exploiting the unique strength of each independent model through model fusion to capture different patterns in the data [14–16]. Specifically, the fusion of classical time series regression models with neural networks indicates the validity of the hybrid approach involving linear and nonlinear components in forecast tasks [17, 18]. In addition, there are studies focusing on optimizing the weight pattern of fusion strategies to produce enhancements in the overall forecast fitting [14, 15, 18].

Relative to general epidemics, the restrictions of available data require dengue forecast models to have the ability to learn valid information from limited features. Although meteorological factors can be used to predict the epidemic situation, taking them as principal characteristic variables and ignoring other disease-related features lack robustness and interpretability [3, 19]. Given the singleness of the expression ability of meteorological characteristics, some studies supplemented the vector surveillance data and verified the potential of mosquito-borne features to improve the predictive ability for dengue risk [5, 20]. Considering that mosquito abundance as a driver of dengue can provide a sufficient window period for early prevention of dengue outbreaks [4], some studies are dedicated to the forecast of mosquitoes themselves [21, 22]. However, to the best of our knowledge, there is still a lack of studies linking the high variability of mosquito fluctuations with dengue cases in the spatiotemporal dimension and as predictors of impending dengue risk. [23]

### 2.2. Correlation Analysis

Although the significance of spatiotemporal associations between mosquitoes and dengue in forecasting dengue risk is not emphasized, some studies analyzed the correlation in terms of time or space [4, 6, 7, 10, 11].

Various approaches such as cross-correlation function and regression modeling were adopted to depict the temporal correlation between dengue risk and larval indices, which validated that mosquito abundance was the determinant of dengue [4, 7, 10]. The potential of larval indices as an early warning signal for dengue was estimated by receiver operating characteristic (ROC) curves without demonstrating its availability in actual forecast scenarios by specific modeling.

Relative to temporal correlation analysis, it is of great significance to assess the spatial distribution pattern of dengue cases and mosquito abundance. In addition to visual analytical modeling of epidemic transmission dynamics [24, 25], several studies are aimed at exploring the spatial dependence of variables, including Pearson correlation analysis and Moran's index [11, 26]. However, Moran's index as a spatial autocorrelation indicator only measures the neighborhood dependence of univariate and is not utilized to analyze the multivariate spatial association that considers the cross-correlation among variables.

## 3. Preliminaries

### 3.1. Problem Formulation

We formalize the aggregation pattern of dengue risk as a spatiotemporal structure diagram shown in Figure 1, where each time slice *t* covers a spatial graph *G* = (*V*, *A*) including grid node set *V* of cases and vectors, and adjacency matrix *A* ∈ ℝ^*N*×*N*^ with grid node number *N*. The mathematical notations are shown in Notations. We assume a time series of length *T* and generate time-ordered records of case numbers and larval indices, denoted as *x*_*t*_ ∈ ℝ^*D*×*N*^(*t* = 1, 2, ⋯, *T*) with each record *x*_*t*_ containing *D* features on *N* nodes. *x*_*t*_^*d*,*i*^ denotes the observed value of feature *d* for node *i* at *t*-th time step. Thus the forecast issue is formulated as given the dengue data *X* = (*x*_1_, *x*_2_, ⋯, *x*_**τ**_) in *τ* time steps to predict case numbers ${\hat{y}}_{\tau +\gamma }\in \mathbb{R}$ with the forecast window length *γ*.

### 3.2. Data Preprocessing

Data were collected according to dengue cases, mosquito vectors, and geographic information and uploaded to the monitoring center by relevant personnel as shown in Figure 2. The cases were divided by source region adopting the regular matching approach. Due to the clutter of raw data, data cleaning is required before feature extraction, including time slice segmentation based on timestamps and grouping in line with grid nodes. The extraction approach of mosquito density is to select more than 400 households distributed in four streets to check all water containers within 5 meters outdoor and then calculate larval indices as shown in (1). Thereinto, pos_con and pos_house are the number of mosquito larva-positive containers and households, and sum_con and inv_house indicate the total amount of investigated containers and households.

(1) $$\begin{array}{c} \text{BI}=\frac{\text{pos}\_\text{con}}{\text{inv}\_\text{house}}*100,\\ \text{CI}=\frac{\text{pos}\_\text{con}}{\text{sum}\_\text{con}}*100,\\ \text{HI}=\frac{\text{pos}\_\text{house}}{\text{inv}\_\text{house}}*100. \end{array}$$

We follow up with data filtering and normalization to eliminate outliers after data segmentation. Affected by the sampling frequency of mosquito vector monitoring, there are missing values in time series data that need to be filled. Missing value processing adopts the surrounding mean filling method to conduct the calculation based on the weighted average of the nearby data. Further, forward-filling is adopted, assuming that missing values are the same as variable observations at the previous time step, taking into account the temporal correlation of time series data. After preprocessing the data according to Figure 2, feature extraction is carried out by components separately.

## 4. Methods

Taking the transmission of dengue is exposed by spatiotemporal factors, we propose STCFM to characterize temporal trends and spatial distributions based on considering statistical properties and integrating them for forecast tasks. Specifically, it is discussed from the following three components.

1. Since the observations of dengue cases exhibited autocorrelation, we adopted the attribute representation in general statistical analysis to construct the statistical component model. Analyze multidimensional statistical properties of dengue cases at independent time steps
2. Considering the lag cross-correlation between dengue risk and mosquito abundance, we constructed a temporal component model with three subcomponents that could depict the short-, mid-, and long-period characteristics of time series
3. We assessed multivariate spatial dependencies of dengue risk and mosquito abundance based on spatial aggregation analysis and constructed the spatial component model with correlation metrics as additional features

The model structure is shown in Figure 3.

### 4.1. Statistics Component Model

Given that risk outbreaks of dengue are observed to be autocorrelated, we propose a statistics component model to characterize the statistical properties of dengue case sequences. The transmission of dengue is affected by the latency, so we define a time window as the length of the incubation period and calculate the statistical properties in the window, including Sum, Incr, Mean, Med, Max, and Min. Moreover, the same period last year (SPLY) was added as a feature attribute due to the observed seasonality of dengue outbreaks. Connecting the above features, the input variables of the statistical component model are constructed as follows:

(2) $$\begin{array}{c} S_{t}=\text{Su}{\text{m}}_{t}\circ \text{Inc}{\text{r}}_{t}\circ \text{Mea}{\text{n}}_{t}\circ \text{Me}{\text{d}}_{t}\circ \text{Ma}{\text{x}}_{t}\circ \text{Mi}{\text{n}}_{t}\circ \text{SPL}{\text{Y}}_{t}, \end{array}$$

where the subscript denotes the time step. Statistical property forecast adopts LSTM (long short-term memory) model applicable for sequence learning tasks involving temporal order recognition in noisy input streams [27].

The structure shown in Figure 4 exhibits the information flow in the memory unit, where the hidden cell state *C* can save long-interval related information to alleviate the time dependence issue to a certain extent. The LSTM model has three inputs in the form, *x*_*t*_ is the current sequence data, *h*_*t*−1_ is the output of the previous unit, and *C*_*t*−1_ denotes the memory of the previous moment. The training of the hidden layer is to process input vectors through forget, input, and output gates in LSTM cells to generate the output value *H*_*t*_ and update the memory *C*_*t*_. Update functions are as follows:

(3) $$\begin{array}{c} f_{t}=\sigma \left(W_{f}h_{t-1}+U_{f}x_{t}+b_{f}\right), \end{array}$$

(4) $$\begin{array}{c} i_{t}=\sigma \left(W_{i}h_{t-1}+U_{i}x_{t}+b_{i}\right), \end{array}$$

(5) $$\begin{array}{c} {\tilde{C}}_{t}=\tanh\left(W_{c}h_{t-1}+U_{c}x_{t}+b_{c}\right), \end{array}$$

(6) $$\begin{array}{c} C_{t}=f_{t}⊙C_{t-1}+i_{t}⊙{\tilde{C}}_{t}, \end{array}$$

(7) $$\begin{array}{c} o_{t}=\sigma \left(W_{o}h_{t-1}+U_{o}x_{t}+b_{o}\right), \end{array}$$

(8) $$\begin{array}{c} h_{t}=o_{t}⊙\text{tanh}\left(C_{t}\right). \end{array}$$

As the output of the forget gate, *f*_*t*_ determines the forgetting probability of the hidden cell state in the previous layer through the nonlinear activation function *σ* (sigmoid) with the value in [0,1]. *W* ∈ ℝ^*H*×*H*^ and *U* ∈ ℝ^*H*×*D*^ denote the coefficient matrix of hidden states and input vectors, where *H* is the number of hidden units, and *b* refers to the bias parameter. The input gate consists of (4) and (5) to selectively store new information in the cell state. *i*_*t*_ and *f*_*t*_ act on the previous state *C*_*t*−1_ and the candidate vector ${\tilde{C}}_{t}$ obtained by tanh activation at the current moment, respectively, as weight parameters to update the cell state *C*_*t*_ as (6), where ⊙ is Hadamard product. *h*_*t*_ is updated by (8) with the output gate *o*_*t*_ obtained by (7) that determines the portion of the cell state *C*_*t*_ activated by tanh. The output layer computes the output value ${\hat{y}}_{t}$ through weighted connections of the hidden layer series *h*_1_, *h*_2_, ⋯, *h*_*t*_.

### 4.2. Temporal Component Model

Generally, even if time series data has evident periodic characteristics, it presents stochastic variations, which are difficult to represent by independent models. Embedding temporal information into forecast models as explanatory factors rather than casual factors to learn the feature trends at different stages is required to be explored, and verifiable interpretability needs to be provided to guarantee the credibility of the model. The majority of current time series forecast models rely only on historical segments adjacent to the forecast period, which are sensitive to missing data and lead to a lack of robustness in forecasting [28]. Given the seasonality of dengue outbreaks, periodic information contained in historical data may not be reflected in recent data. We propose a solution that combines short-, mid-, and long-period features, which divide time series into three stages and model them separately to flexibly capture the impact of multivariate temporal dependencies on forecasting tasks [28]. Specifically, we construct a temporal component model with three subcomponents to depict the feature in short-, mid-, and long-periods, and the corresponding temporal segments are denoted as *T*_*s*_, *T*_*m*_, *T*_*l*_, as shown in Figure 5.

Considering that the epidemic outbreak is affected by the incubation, we define the adjacent time segment of the forecast target as *T*_*s*_, covering the length of the incubation period (14 days). Additionally, the outbreak peak of dengue is observed to exhibit seasonal variation, so *T*_*l*_ is defined as the time segment one year before the forecast target to model the variation pattern with an annual cycle. Unlike *T*_*s*_ and *T*_*l*_, *T*_*m*_ as the midterm segment requires temporal correlation analysis to determine the appropriate value, which cannot be obtained simply by observation or experience. Since dengue is transmitted through dense populations established by mosquitoes, larval indices can serve as an early warning signal to explain dengue outbreaks [4]. To reasonably introduce larval indices into predictors, we conducted temporal lag correlation analysis on monthly data collected from mosquito-borne infectious disease surveillance reports and found a lag relationship between vector density index and dengue case numbers. Specifically, we assessed the dynamic variation of fitted correlations between time series with time through the temporal lag cross-correlation function. We select Spearman's rank correlation coefficient, commonly considered a metric of monotonic correlation, to quantify the interseries correlation with the lag of *k*‐th time step. Suppose the time series *X*_1_, ⋯, *X*_*T*_ and *Y*_1_, ⋯, *Y*_*T*_ denote larval indices and dengue case numbers. The lag correlation between *X*_*t*_ and *Y*_*t*+*k*_ is defined as follows:

(9) $$\begin{array}{c} \rho_{XY}\left(k\right)=\left\{\begin{array}{cc} 1-\frac{6\sum_{t=1}^{T-k}{\left({\tilde{Y}}_{t+k}-{\tilde{X}}_{t}\right)}^{2}}{\left(T-k\right)\left({\left(T-k\right)}^{2}-1\right)}, & \text{if}k\geq 0,\\ 1-\frac{6\sum_{t=1-k}^{T}{\left({\tilde{Y}}_{t+k}-{\tilde{X}}_{t}\right)}^{2}}{\left(T+k\right)\left({\left(T+k\right)}^{2}-1\right)}, & \text{if}k<0, \end{array}\right. \end{array}$$

where ${\tilde{Y}}_{t+k}$ and ${\tilde{X}}_{t}$ denote the position of *Y*_*t*+*k*_ and *X*_*t*_ after sorting separately, and *T* represents the length of the time series as shown in Notations. The value is between -1 and 1, with the absolute value indicating the correlation. The results illustrated that dengue cases exhibited a significant positive correlation with larval indices lagged by one-month period (*r* = 0.638, *p* < 0.001), which is used to determine *T*_*m*_ to build an midperiod temporal model. Based on the above analysis, we intercepted *T*_*s*_, *T*_*m*_, and *T*_*l*_ to constrain feature sequences in different periods and maintain the length consistency. The specific definitions are illustrated in Figure 5. We train temporal correlation features through the LSTM model, where each subcomponent shares the neural network structure. The significant superiority lies in that it can use contextual information when mapping input and output sequences to solve the vanishing gradient problem for long temporal lag tasks [29].

### 4.3. Spatial Component Model

Lag is generally expounded in terms of time, whereas spatial lag measures the spatial dependence of variables according to topological associations. Specifically, it represents the local influence of surrounding areas on the current region in a fine-grained manner through the weighted average observations of variables in the neighbors. The Moran index is a quantitative study of aggregation phenomena in different geographic locations based on spatial lag, usually limited to spatial autocorrelation analysis [11]. Instead, our work estimates bivariate spatial cross-correlation coefficients between larval indices and dengue cases to measure the spatial dependence among different variables and explore its potential as a predictor. Specifically, we extend the concept of local spatial autocorrelation to the binary spatial correlation issue with the essential difference that the spatial lag calculation under bivariate pertains to different variables. In addition to topological associations of observations, it also focuses on cross-correlations [30].

We partition the geographic layer into *N* grids and extract spatial factors according to the spatial distribution of cases in the actual scenario. Extend the spatial lag to a bivariate dimensional context by analyzing the relevance between dengue cases *y* at region *i* and larval indices *x* at the adjacent region *j* as follows: *L*_*t*_(*y*_*i*_) = ∑_*j*_^*N*^*a*_*ij*_*x*_*j*_, where *y*_*i*_ and *x*_*j*_ are both normalized. Spatial correlation within the general definition does not account for different variables in the same region but requires to be considered in our context. In this regard, we consider the node itself through self-connection and realize the calculation of intrinsic correlation. The specific method is to obtain the adjacency matrix *A* as the spatial weight value according to the geographical distribution of the region, where *a*_*ij*_ is 1 indicates that regions *i* and *j* are adjacents, and 0 is not. Besides, *A* is updated by *A* + *I*_*N*_ that added self-connection.

(10) $$\begin{array}{c} A=A+I_{N}=\left[\begin{array}{cccc} a_{11} & a_{12} & \cdots & a_{1n}\\ a_{21} & a_{22} & \cdots & a_{2n}\\ \vdots & \vdots & \ddots & \vdots \\ a_{n1} & a_{n2} & \cdots & a_{nn} \end{array}\right]+\left[\begin{array}{cccc} 1 & 0 & \cdots & 0\\ 0 & 1 & \cdots & 0\\ \vdots & \vdots & \ddots & \vdots \\ 0 & 0 & \cdots & 1 \end{array}\right]. \end{array}$$

The spatial cross-correlation pattern between dengue cases and mosquito abundance was then calculated by the bivariate local Moran's index as follows:

(11) $$\begin{array}{c} I_{i}=C{\tilde{y}}_{i}\overset{N}{\underset{j}{\sum }}a_{ij}{\tilde{x}}_{j}, \end{array}$$

where ${\tilde{x}}_{i}=x_{i}-\bar{x}$, ${\tilde{y}}_{j}=y_{j}-\bar{y}$, and *C* is for standardization. In the context of this work, *I*_*i*_ > 0 denotes there was a positive spatial cross-correlation between cases in the region *i* and mosquito abundance in the surrounding area, and $\sum_{j}^{N}a_{ij}{\tilde{x}}_{j}$ indicates the corresponding spatial lag value. A bivariate Moran scatter plot is optimized in the form of a bubble chart to visualize the spatial lag relationship, as shown in Figure 6(a), where the abscissa is the ${\tilde{y}}_{i}$ value of case and the ordinate indicates the spatial lag in the context of larval indices. The product of abscissa and ordinate maps the bivariate local Moran's index. And the size of bubble data points is determined by the number of regions corresponding to this value. The fitted trend line demonstrated a positive spatial correlation between dengue cases and larval indices. Mapping the quadrants in the scatter plot on the geographical location in the form of a color block diagram is the Moran Map in Figure 6(b), and its specific mapping rules are depicted in the legend. Moran map intuitively exhibits the spatial correlation of variables in different geographic locations.

Spatial lag values and bivariate local Moran's index obtained from multivariate spatial correlation analysis were added as features to the spatial component model. It is worth mentioning that the spatial correlation metric among three larval indices (BI, CI, and HI) and dengue cases has high pertinence. Considering the impact of redundant inputs on the robustness of neural networks, we use BI as the proxy of mosquito abundance features for spatial correlation calculation. We choose ConvLSTM [31] as the spatial component model to learn the spatial dependencies of dengue cases and mosquito abundance. ConvLSTM is based on LSTM structure but adopts convolution instead of state-state full connection mode, which further extracts spatial information compared to LSTM, as shown in Figure 7. Specifically, the input is regarded as an eigenvector distributed on the spatial grid, and ConvLSTM determines the future state of the current spatial node by convolution operations on the past states of other grid cells. The update equations are as follows:

(12) $$\begin{array}{c} f_{t}=\sigma \left(W_{hf}*h_{t-1}+W_{xf}*x_{t}+W_{cf}⊙C_{t-1}+b_{f}\right),\\ i_{t}=\sigma \left(W_{hi}*h_{t-1}+W_{xi}*x_{t}+W_{ci}⊙C_{t-1}+b_{i}\right),\\ C_{t}=f_{t}⊙C_{t-1}+i_{t}⊙\text{tanh}\left(W_{hc}*h_{t-1}+W_{xc}*x_{t}+b_{c}\right),\\ o_{t}=\sigma \left(W_{ho}*H_{t-1}+W_{xo}*x_{t}+W_{co}⊙C_{t}+b_{o}\right),\\ h_{t}=o_{t}⊙\text{tanh}\left(C_{t}\right), \end{array}$$

where ∗ denotes the convolution operation and ⊙ denotes the Hadamard product. It can be interpreted that the quantity of dengue cases in the designated region is not merely related to the current region but also affected by other areas.

### 4.4. Fusion Strategy

A single decision model tends to ignore the indeterminacy, and complexity of data and is not universal. The fusion methodology exploits the unique preponderances of component models and theoretically be capable of improving the forecast performance of time series in contrast with independent models. Considering the characteristics that different models recognize different data patterns in practical scenarios, this study utilizes an ensemble learning strategy to fuse *N* learners to train spatiotemporal features.

Due to the heterogeneity of component learners, this work introduces the Stacking ensemble framework with two-tier architecture to model component learners. Specifically, the outputs obtained by the primary learner based on original samples are used as the input features of the secondary model, and the metalearner is utilized in the second layer instead of voting or averaging to fuse the strength of the independent model and fit the regression results. Compared with Bagging and Boosting algorithms in ensemble learning, the Stacking method enhances the expressiveness and generalization and reduces bias and variance. And relative to the BMA combination strategy being sensitive to model approximation error, the advantage of Stacking is reflected in robustness [32].

To integrate the superiority of each submodel to improve performance, component learners should be discriminative and accurate. By constructing statistics, temporal, and spatial components, we simultaneously capture the characteristics of the three dimensions in statistical properties, temporal trends, and spatial distributions. Considering the influence of metalearner on the generalization performance, we select the commonly used multiple linear regression (MLR) model to seek the optimal function by minimizing the sum of squared errors. And on account of the temporal dependence, forward chain cross-validation was adopted to reduce the risk of overfitting. Suppose the output sequence $\hat{y}={\left[{\overset{\wedge }{y}}_{1},{\overset{\wedge }{y}}_{2},\cdots ,{\overset{\wedge }{y}}_{T}\right]}^{⊤}$, and *T* denotes the length of the time series. For output ${\hat{y}}_{t}\in \mathbb{R}$, multiple linear regression is represented by the following:

(13) $$\begin{array}{c} {\hat{y}}_{t}=w_{0}+w_{1}{\hat{y}}_{t}^{1}+w_{2}{\hat{y}}_{t}^{2}+\cdots +w_{n}{\hat{y}}_{t}^{n}, \end{array}$$

where a total of *n* forecast models, ${\hat{y}}_{t}^{i}$ denotes the forecast result of the *i*-th model at time *t*, and *w*_*i*_ measures the impact of different component models on the forecast results.

## 5. Case Study

We conducted comparative experiments on real-world dengue datasets to verify the effectiveness of the proposed model. The remainder of this section presents the dataset and implementation details and a comparative analysis of the empirical results.

### 5.1. Datasets

The Lancang-Mekong region, including Yunnan Province, has a high incidence of dengue due to its subtropical climate, which is prone to breeding mosquitoes. The surveillance sites deployed in Yunnan Province and surrounding areas collected and recorded dengue and mosquito data through relevant personnel, covering the Jinghong region with the period spanning 2013 to 2019. We constructed the dataset as samples with geographic location information of 14-day intervals, including features of statistical properties, temporal trends, and spatial distributions that accompany time windows.

Due to the temporal sequence sensitivity, the dataset was split into the training set, validation set, and test set in a 6 : 2 : 2 ratio in chronological order. It is worth noting that, in contrast to the majority of models that predict in an in-sample way, we adopt out-of-sample modes to conduct retrospective analysis and forecast to estimate performance, which has robust interpretability for possible overfitting issues.

### 5.2. Implementation Details and Baselines

We contrast the proposed forecast model against the following baselines to verify the model performance.

- *Historical Average (HA)*. Use the average of observations from adjacent historical segments as the predicted value.
- *ARIMA*. ARIMA(*p*, *d*, *q*) model [33] in the Box-Jenkins method is the benchmark for time series forecast, where *p*, *d*, and *q* are determined by minimizing the Akaike information criterion (AIC).
- *SVR*. Support vector regression (SVR) is a supervised learning method for regression analysis [34]. We select the radial basis function (RBF) kernel that conforms to Mercer's theorem for nonlinear modeling in time series prediction scenarios.
- *XGBoost*. Extreme gradient boosting [35] is an optimized ensemble tree model that implements parallel forecast algorithms under the gradient boosting decision tree framework.
- *CNN*. Convolutional neural networks (CNN) [36] are feedforward neural networks with deep structure composed of convolutional layers and pooling layers.
- *LSTM*. A long short-term memory network [29] consisting of forget gates, input gates, and output gates can learn the long-term dependency of time series.

We implement the above candidate models through the sklearn library and the TensorFlow framework. For STCFM, we set the hidden units of LSTM to 32 with a batch size of 8. The loss function is set to mean squared error, and the Adam optimizer is utilized [37] with the learning rate set to 0.001. The spatial component model consists of three layers of ConvLSTM with 32 filters for the convolutional layers and a kernel size set to 3. The grid spacing in the spatial dimension is partitioned according to the actual distance of 5 kilometers, and the temporal window length is set to 14 days through the time step parameter.

### 5.3. Evaluation Criteria

Two general metrics are adopted to evaluate the performance of candidate models.

1. *Root Mean Square Error (RMSE)*. RMSE is used to assess the discrepancy between the predictive value $\hat{y}$ and the corresponding true value *y*, as closer RMSE to 0, indicating a better forecast performance. The calculation formula is

(14) $$\begin{array}{c} \text{RMSE}=\sqrt{\frac{1}{T}\overset{T}{\underset{i=1}{\sum }}{\left({\overset{\wedge }{y}}_{i}-y_{i}\right)}^{2}} \end{array}$$

(2) *Coefficient of Determination* (*R*^2^). *R*^2^ is utilized to measure the goodness of fit of the forecast model with the value range of [0,1] and calculated as follows. The closer *R*^2^ is to 1, the more accurate the forecast

(15) $$\begin{array}{c} R^{2}=1-\frac{\sum_{i=1}^{T}{\left({\overset{\wedge }{y}}_{i}-y_{i}\right)}^{2}}{\sum_{i=1}^{T}{\left({\bar{y}}_{i}-y_{i}\right)}^{2}} \end{array}$$

### 5.4. Empirical Results

We compared STCFM with six candidate models on the dengue dataset, where the forecast window is set to day and week, and the experimental results are shown in Table 1. The results illustrate that STCFM achieves optimum performance under both evaluation criteria regardless of the forecast step length. Compared with deep learning algorithms, the poor performance of general machine learning approaches on the dengue risk forecast task stems from limited modeling capabilities. STCFM outperforms all candidate models due to its simultaneous consideration of temporal correlation and spatial dependence.

The forecast performance of HA is acceptable compared to other machine learning approaches because of the imbalanced nature of dengue data. It can be interpreted that HA has a steady forecast effect in sequence stationary periods with a higher proportion. But it only learns the information of adjacent historical segments, resulting in low forecast accuracy for the risk outbreak period with volatility. Given the uncertainty of dengue risk due to multiple factors, deep learning algorithms with higher flexibility are more suitable, as shown by CNN and LSTM in Table 1. Compared to the two best performing candidate models, CNN and LSTM, STCFM achieves 18.2% and 9.8% relative improvement on *R*^2^ in the week metric, 13.7% and 5.0% in the day metric. It attributes to the mining of spatiotemporal dependencies by the spatiotemporal component fusion strategy, which introduces the convolution operation of CNN while exploiting the long memory capability of LSTM to achieve the purpose of capturing spatiotemporal features. We further adopt *R*^2^ to assess the performance variation of each approach with increasing forecast step length, as shown in Figure 8. It can be seen from the figure that the goodness of fit of candidate models decreases with the increase of forecast time. STCFM outperforms the baselines mentioned above and exhibits insensitivity to the variation of forecast step length, implying that STCFM has potential for long-term prediction tasks.

In addition, to analyze the effectiveness of the spatiotemporal feature factors added in STCFM and the necessity of component fusion, we conduct comparative experiments from the feature dimension to verify the optimal combination pattern of features. Specifically, we separately analyzed the forecast results of the statistical feature sequences of dengue cases and the multivariate feature sequence with temporal lag periods and spatial lag coefficients. And further, explore the impact of component fusion and forecast step length on the forecast performance. We measure the forecast performance of different feature combinations with RMSE and *R*^2^ as the forecast step length increases and shows in Figures 9(a) and 9(b), respectively. The results intuitively exhibit that the introduction of temporal and spatial factors enhances the ability of the model to forecast dengue risk. It confirms that the explicit modeling of data in different periods by temporal component strengthened mining utility for temporal features and represents the multiscale variation patterns of dengue risk and mosquito abundance. Further, introducing spatial correlation metrics into spatial components constructs valid feature representations and improves forecast performance with ConvLSTM that captures spatial correlations. The above results validate that we have obtained an effective spatiotemporal feature representation using a reasonable correlation analysis method. And utilizing them as predictors to solve the issue of dengue risk forecast is a creditable attempt.

## 6. Conclusions

In this paper, we propose STCFM to fuse spatiotemporal components for dengue risk forecast. Specifically, we first construct the statistics component model based on statistical analysis variables of dengue data. Then, considering the influence of mosquito-borne factors on dengue transmission, the spatiotemporal lags obtained by correlation analysis were drawn into multivariate feature sequences to construct spatial and temporal components. The temporal component model conducts multiscale modeling of time dependencies by capturing short-period, mid-period, and long-period historical variations of data, enhancing the predictive capacity because of relevant temporal segments with potential impact. The spatial component model adopts spatial correlation metrics as additional predictors and utilizes ConvLSTM to train spatial features based on the positive correlation of data in the spatial dimension. Finally, all components are fused through the stacking strategy in ensemble learning.

Experimental results illustrate that STCFM outperforms the candidate models, and the involved spatiotemporal feature learning approaches and component fusion strategies can be extended to data analysis and forecast issues in other domains. In future work, we expect to develop a general forecast visualization framework to simultaneously visualize feature representations and the spatiotemporal transfer process of events, enabling optimization of the model structure by providing various valuable visual information.

## Figures and Tables

**Figure 1:** Abstract schematic diagram of spatiotemporal dependence.

**Figure 2:** Data preprocessing flowchart.

**Figure 3:** Model component structure of STCFM.

**Figure 4:** LSTM framework.

**Figure 5:** Multiscale time series segment construction.

**Figure 6:** Multivariate spatial correlation visualization.

**Figure 7:** ConvLSTM framework.

**Figure 8:** Variation in *R*^2^ for different candidate models as the forecast step length increases.

**Figure 9:** Performance comparison of different component combinations.

**Table 1:** Forecast performance comparison with different models.

Model	RMSE (week)	*R* ^2^ (week)	RMSE (day)	*R* ^2^ (day)
HA	48.64	0.58	6.05	0.70
ARIMA	69.02	0.18	10.16	0.19
SVR	58.36	0.39	7.17	0.58
XGBoost	48.99	0.57	7.05	0.59
CNN	43.44	0.66	5.72	0.73
LSTM	42.18	0.68	5.61	0.74
STCFM	34.88	0.78	4.65	0.83

## Data Availability

The raw data used to support the findings of this study have not been made available because they contain information that could compromise the privacy of research participants.

## Notations

*x*: Input data
*y*: Observed value of forecast target
$\hat{y}$: Forecast result
*τ*: Time series length
*γ*: Forecast window length
*T*, *N*, *D*: Dimension in temporal, spatial, and feature
*S*_*t*_ ∈ ℝ^*D*^: Statistical property features at *t*-th time step
*T*_*s*_, *T*_*m*_, *T*_*l*_: Time series segment construction in short, mid, long period
*A* ∈ ℝ^*N*×*N*^: Adjacency matrix
*L*_*t*_ ∈ ℝ^*N*^: Spatial lag at *t*-th time step
*I*_*t*_ ∈ ℝ^*N*^: Bivariate local Moran's index at *t*-th time step.
